# Interactive Mode of Visual Communication Based on Information Visualization Theory

**DOI:** 10.1155/2022/4482669

**Published:** 2022-07-31

**Authors:** Xiaoke He

**Affiliations:** Jiangxi Modern Polytechnic College, Nanchang 330095, China

## Abstract

In the modern environment, visual communication design has become a comprehensive subject that combines technology and art. The development of various technologies has promoted the emergence of new design art forms, and at the same time, it has also promoted the change of design concepts and thinking modes. Visual representation, as a representation practice to express the meaning of information in the form of visual symbols, is a method and means to realize information visualization. Based on visual interface design, this article takes interactivity and user experience as innovation points and digs into the design process of interactive information visualization to achieve the purpose of information transmission. By analyzing the cognitive tasks of users in each stage of visual thinking activities in visual terminals, this article proposes to optimize the interactive design of visual communication from the key points of attention, consciousness, and memory. In order to verify the feasibility of the interactive mode of visual communication based on information visualization theory, this article has carried out several comparative experiments with different models. Experimental results show that this algorithm has a faster convergence speed and a greater generalization ability, the accuracy of the algorithm reaches 96.03%, and the highest evaluation of user satisfaction is 95.93%. The interactive mode of visual communication in this article can provide means and reference value for the development direction of visual communication design.

## 1. Introduction

Computer science was the first field to use visualization. It entails transforming a substance into a medium that can be seen with the eyes, that is, the object can be seen and understood through the eyes of the audience [1]. Its goal is to improve the audience's information knowledge and comprehension. In the field of computer graphics, information visualization is a significant accomplishment. Information visualization has long been thought of as a method and tool for helping people understand and analyze large amounts of data. The data age is currently in full swing, and humans are confronted with not only “anything is possible,” but also unprecedented challenges [2]. Visualization technology has been pushed from the laboratory to a broad terminal market as information visualization has gradually branched out from scientific visualization. The research will focus on the analysis of information experience and the availability of information services against the backdrop of the information age. Information visualization is a new subject field that combines multidisciplinary theories and methods from a variety of disciplines, including communication, psychology, statistics, and design [3]. Information visualization typically focuses on assisting expert users in performing complex data exploration and analysis tasks as efficiently and effectively as possible, thanks to its historical roots in scientific reasoning, computer graphics, and algorithm optimization. This advanced data visualization technique is frequently regarded as a scientific tool [4]. At the moment, simply improving visualization quality through advanced technical means is insufficient to meet users' information needs. In order to improve information visualization more comprehensively, it is necessary to fully comprehend users' cognitive processes from perceptual experience to rational thinking.

The research object of information visualization can be divided into three aspects as an interdisciplinary field: data, visualization technology, and visualization performance [5]. People in the information age not only passively accept information, but also actively produce and disseminate it, resulting in a shift in their visual concepts. Image and symbolic information provide obvious visual pleasure to the audience, which provides a good audience foundation for the design and communication of visual communication [6]. Humans organize various visual elements such as words, images, colors, and other elements to achieve the dissemination of public information through visual communication design. It is a type of design that uses visuals to communicate. Visual communication is the process by which the designer transforms ideas and concepts into visual symbols, whereas visual communication is the process by which the receiver transforms ideas and concepts into visual symbols. Visual communication design is a type of design that communicates through visual symbols. The sender of information is the designer, and the receiver of information is the object of communication [7]. An urgent problem is how to make visualization technology better serve information users through a visual communication scheme, make information users understand and process information more easily, and improve the interactive effect of visual communication [8]. Visual representation design of information refers to a designer's visual representation design of information based on the subject of information visualization, using visual communication design knowledge, in order to make the audience easily obtain effective information in the era of big data and achieve maximum dissemination of information. Based on the information visualization theory, this article makes an in-depth study on the interactive mode of visual communication, and its innovations are as follows:

1. Based on the existing theoretical basis of information visualization and visual communication, this article studies the relationship among information visualization, visual representation, and visual communication design and analyzes the communication mechanism of visual representation of information visualization. In the application innovation of dynamic visual innovation and multisensory interactive experience in visual communication design, some typical cases under new technologies are used for research, trying to explore new ideas and methods through case analysis.
2. Based on the existing research results, this article puts forward new views, discusses the visual cognitive representation of information visualization, and broadens the research field of information visualization. According to the existing mode of thinking, combined with our own practice, a systematic design method of visual communication of information visualization is constructed. The effectiveness of this method is verified by experiments, and the superiority of dynamic visual communication in information dissemination is analyzed. In the future, visual communication design in other fields can provide a reference basis.

This article's research content and structure are as follows: Section 1 introduces the article's research context, significance, and organizational structure. Section 2 is primarily a summary and review of relevant domestic and international literature. It also introduces the research and innovation methods used in this article, which are based on these related literatures. Section 3 focuses on information visualization theory and related issues of visual communication interaction mode as well as the interactive information visualization design process. Section 4 details on the experimental analysis. The actual test is carried out in this section, and the test results are obtained, based on the relevant data. The algorithm's performance is evaluated in comparison to the experimental results of other methods. Section 5 concludes the study. This section primarily summarizes the research's main points and findings, summarizes the research conclusions, and suggests future research directions.

## 2. Related Works

Information visual design is a unique discipline that cuts across many industries and is a design category with a wide range of applications. Nowadays, relevant researchers in the field of information visualization have their own unique knowledge and understanding from their respective perspectives as well as a level of depth. Simultaneously, as the vocabulary of media grew, many design firms and avant-garde designers began to experiment with digital multimedia to express creativity and convey information. Visual communication design, as part of the creative field, is attracting increasing attention from all walks of life, playing an increasingly important role in people's lives, and defining the function of information transmission.

Papasarantou et al. examined the often-overlooked appeal of visual appeal in information visualization and discussed the broader role of emphasizing visual communication design principles in the design process [9]. Vera believed that improving the efficiency of visual thinking in processing information and reducing the cognitive load in this process can allow more cognitive costs to be allocated to later abstract understanding and decision-making. Therefore, they conducted research on finding ways to optimize the design of information visualization by understanding the characteristics of visual thinking activities [10]. In order to further understand and engage in scientific information visualization and visual communication design methods, Wu et al. proposed a mutual learning strategy of art and practice [11]. Combined with the development characteristics of information visualization under the background of experience economy, Li and Liu et al. explored solutions to improve the quality of visualization services from the perspective of information users and provided useful suggestions for the research of information visualization in visual communication design and visual effect evaluation [12]. Kosara and Mackinlay used a large number of cases to conduct an in-depth exploration of the practical innovation of visual communication design, thus confirming the two main visual expressions of visual language in new media—one is dynamic and the other is multisensory humanization of interaction [13]. Winstel pointed out that the visual communication design under information technology should not only stay in the traditional design under the influence of technology, but should focus on the “new communication” and “new language” of visual design, and new forms of expression and specific applications in new media are studied in-depth [14]. Compared with other disciplines, visual communication design occupies a pivotal position in information design by Pfeffer. The communication of visual graphics vocabulary is the key to information design and the most basic requirement of visual information construction. On this basis, with the expansion of the application field of information design, its design concept affects business planning, cultural construction, and audience visual interaction experience [15]. Reif et al. obtained the commonality and individuality of digital visual communication design and print design through the comparative analysis of digital visual communication design; and then combined with examples to analyze the immaterial, interactive, and multidimensional language characteristics and dynamics of digital visual communication design, multimedia, and interactive communication characteristics [16]. Haustein et al. took visual communication as the main body of their research and explored the communication mechanism of visual representation of information visualization and the corresponding design method of visual communication of information visualization [17]. Estrada et al. believed that the current design forms for information dissemination only pay too much attention to design symbols, ignoring the psychological needs of the audience and the process of information dissemination, resulting in the inability to maximize the dissemination of information [18]. Han and Deng focused on new media and visual communication design and analyzed the occurrence of new media and its characteristics of the times. At the same time, the connotation and development process of visual communication design are explained in simple terms, and it is concluded that the change of media technology is the main reason for the evolution of visual communication design [19].

In this article, some viewpoints and ideas are put forward based on previous studies on visual communication. On the basis of visual interface design, and taking interactivity and user experience as innovation points, the design process of interactive information visualization is deeply explored. Combining theory with practice, this article explores a systematic design method of visual representation of information visualization. According to the application of design thinking and design methods, the simulation experiment is carried out, and all kinds of boring data information are presented through visual symbols, which eliminates the obstacles between the public and all kinds of information and improves the effectiveness of visual communication interaction.

## 3. Methodology

### 3.1. Information Visualization Theory and Visual Communication Design

Information is defined as meaningful data that can express the objective facts that the data describe. The data that have been organized and sorted have relevance and have become information, but it remains data for those who are not experts in this field and cannot comprehend the meaning expressed by these data. Information visualization is the use of effective visual expression to assist users in reading, identifying, and interpreting data subjectively in order to provide them with access to critical data. More personalized and customized information visualization works have been published through the Internet platform since the arrival of the experience economy, which not only benefits users' information quality but also poses new challenges to information visualization design. The visualization product should be able to reach the brain via human vision, hearing, touch, and even other senses, and instantly understand a large amount of data [20]. Information visualization emphasizes people's receptivity while also incorporating psychology, visual design, human-computer interaction, business methods, and other disciplines. The symbolic design in the practice of visual representation is the reason why the visual view of information can convey information to the public. The ability of the audience to interpret the meaning of symbols provided by designers determines the effectiveness of information communication. Information communication is ineffective if the audience does not understand the meaning of the symbols.

Information visualization has been adopted by many media and educational, government, and corporate organizations due to its understandable visual form and inherent ability to present complex data. When users contact the information visualization platform, one of the most common cognitive activities is visual thinking. Visual thinking, in contrast to other abstract thinking activities, is based on perceptual experience and can complete a variety of cognitive tasks. The disseminator, receiver, information, and carrier are all involved in the visual representation of information, which is a two-way interaction between coding and decoding in information dissemination. At the same time, the information visualization view is a type of construction, with the representation being the representation that is dependent on the construction, and the construction being the construction that requires representation, all of which combine to form the information visualization view's meaningful communication. Information can be visualized while being read to alleviate the pressure of a “information explosion” caused by a large amount of data. When creating information graphs, the accuracy of information visualization is critical. Before beginning the design, it is necessary to have a solid foundation of theory, science, and technology, and the resulting infographic must be completely accurate. When designing infographics, this is where designers can easily make mistakes. In comparison to large data sets generated by scientific calculations and engineering surveys, information visualization resources are nonphysical and abstract, with no obvious spatial characteristics. The information visualization process and system structure are shown in Figure 1.

With the gradual expansion of the scope of modern design, digital technology and network technology have penetrated into all fields of visual communication design, and the influence and participation of multimedia technology on art and design are getting deeper and deeper, which makes visual communication design step onto a brand-new stage. Information design and graphic design serve different purposes: the former is concerned with “effective information transmission,” while the latter is concerned with “exquisite artistic expression.” The visual effect is more innovative and unique because the image generation technology for information visualization is not complicated, and its expression methods are diverse. Individuals, businesses, and even countries can be clients of information visualization. These forms are important, but the service content is what matters most. Information visualization covers a wide range of disciplines and application fields as an important method in information design. It can be used to solve specific professional problems. The faster and more agile the visual thinking can respond to the input visual information, the more accurate and reasonable the visual communication of information is. Information visualization examines the data visualization presentation results, extracts the hidden value from the data, and assists in making sound decisions. Because this type of decision is not invariable in a constantly updated data environment, information visualization is a continuous process that allows users to discover potential problems and improve the final decision in stages over time. In the visual communication design of information visualization, color serves as a classification and emphasis tool. Color distinguishes primary and secondary relationships and categories. In visual perception, color is the most intuitive, and information can be obtained without using logic.

Computer science research [21, 22] in information visualization mainly focuses on solving users' functional requirements. This technical research can reduce the impact of other problems such as aesthetics or user experience [23]. Visual communication design always takes the audience's acceptance of visual information through their own aesthetic judgment as the ultimate goal, and visual communication design always pursues and yearns for a rational interaction with the audience, thus turning the communication of visual information into effective communication with people. Interaction is a convenient way for users to operate content and its attributes. Interaction is a technology that can easily explain products and make the audience feel relaxed when reading information. The two-way interactive communication mode of visual information makes the new media visual communication design pay more and more attention to the audience's necessity and “participation” in the design. On the contrary, more and more people are looking forward to bringing their ideas and wishes into the design, which promotes the formation of interactive design. As information visualization design is a very wide range of disciplines, in the process of visualization, the application of visual communication design has a transformational impact on the ways and means of attaching importance to teaching and carrying out information visualization research. Graphic symbols account for the largest proportion in information view, which is the soul of visual representation of information. Graphic symbols include pictures, theme graphics, attached icons, charts, and characters. This article analyzes and summarizes the classification of graphics, the effectiveness of attached icons, the model construction of charts, and different types of characters. The more and faster cognitive tasks are accomplished by visual thinking, the more cognitive costs can be allocated to abstract thinking activities, thus improving the efficiency of people's deep understanding of information and making decisions.

### 3.2. Interactive Design of Visual Communication Based on Information Visualization

Graphic symbols are image materials generated by various graphic software, and their visual representation differs from that of words and languages. Graphics, which are the main visual representation symbol in information visualization design, can be copied in large quantities using various methods. Because the main graphic symbol is so closely linked to the information visualization theme, it can be said that the main graphic symbol is the information theme's mapping. Visual communication design in the modern world is interactive design with people that emphasizes the audience's active cognition in the process of receiving information and selectively accepts visual information based on their own aesthetic demands and wishes. The more experience and knowledge an information user has with information acquisition and understanding, the faster and more accurately he can extract the information content he needs from the visual interface and the more effectively he can dig out the connotation and relationship of information and find solutions to problems. Tagged words are concise, clear, and easy-to-understand that appear in the view as expressive keywords. The introduction or explanation of a specific piece of information or a group of related pieces of information is included in descriptive text. The orderly arrangement of some data and information in the information view, which makes the information more intuitive and reduces the audience's visual pressure, is known as organized text. A basic visual model is chosen to express it is “representation.” This step essentially determines the nascent form of the visualization effect, and it is necessary to consider the appropriate representation method based on the data dimensions, such as a list, tree structure, or other methods. The goal of “decoration” is to make information expression simple and clear while also being rich in connotation, practical, and beautiful. To create a logical structure, the information hierarchy must first be divided. After grouping and classifying the data, graphic design is used to convey information of various dimensions, such as category, attribute, degree, orientation, etc., and data of all types and dimensions are sorted according to the information needs of users to highlight the most pressing issues.  Figure 2 depicts an interactive design diagram of visual communication based on information visualization.

Abstract graphic symbols are completely out of the natural form, and it is impossible to extract a specific image from them, so it is necessary for viewers to create graphics with their imagination. Figurative figure is a form that is close to the viewer's daily life and the objective facts. It can reproduce the features of things and is direct, vivid, clear, and easy to identify. Dynamic visual symbols can attract more attention from the audience, which also makes the new media visual communication design not only need to pay attention to the expression form of plane visual elements, but also consider its animation effect in the picture. The difference of visual information determines its “pop-up effect.” The better the pop-up effect, the easier it is to pay attention to screening. Therefore, the target information can be “popped up” from the background or nontarget information by changing the visual features such as color, size, position, and shape. Data mining or statistical methods are used to analyze the data format or put the data in a mathematical environment. Its purpose is to find some rules in a pile of chaotic data, so as to provide organized raw materials for subsequent data representation. Visual representation is the method and way to realize information visualization. It refers to the multi-method of “visualization” for information representation, so that the represented information can be “visualized,” and finally the information can be optimized, so as to promote the public's acceptance and understanding of information, maximize the information dissemination, and innovate the information dissemination process.

If the coordinate of the root node is (*X*_0_, *Y*_0_), the selected radius is *r*; the number of direct child nodes is count. Then the formula for calculating the coordinate (*X*_*i*_, *Y*_*i*_) of the *i*th child node is as follows:

(1) $$\begin{array}{c} X_{i}=X_{0}+r^{*}\cos\left(\frac{2p^{*}i}{\text{count}}\right), \end{array}$$

(2) $$\begin{array}{c} Y_{i}=Y_{0}+r^{*}\sin\left(\frac{2\pi^{*}i}{\text{count}}\right). \end{array}$$

If the coordinate of *A* is (*X*_0_, *Y*_0_), and the included angle of *A* on its concentric circle is initAngle, the formula for calculating the coordinate (*X*_*i*_, *Y*_*i*_) of the *i*th child node in the next layer of *A* is as follows:

(3) $$\begin{array}{c} \text{initAngle}=\arctan\left(\frac{Y_{0}}{X_{0}}\right),\\ X_{i}=X_{0}+r^{*}\cos\left(\text{initAngle}+2p+\frac{i}{\text{count}}\right),\\ Y_{i}=Y_{0}+r^{*}\sin\left(\text{initAngle}+2\pi +\frac{i}{\text{count}}\right). \end{array}$$

It is possible to improve the quality of the user experience by creating a favourable situation. Information visualization design can incorporate materials related to users' knowledge base, life experience, and personal details. The arrow is the most widely used directional symbol in the visual representation design of information visualization, and it has various meanings in various contexts. Computers perform the majority of the design work. The user's status shifts from passive to active in the interactive stage, from acceptance to discovery and consideration. The ability to control and explore data through interface interaction allows them to truly combine computer and human intelligence. The visible part of the user's interface is called the man-machine interface. Communication and operation with the system require a man-machine interface. Under new media technology, it is the most unique design language in visual communication design, and the interactivity of visual communication design has been fully demonstrated in a variety of design practices. Expert users can understand and analyze data at a deeper level thanks to interaction. For obtaining implicit data knowledge, an interface is required. The introduction of a comprehensive digital network has created unprecedented opportunities for interaction and the collection of a wide range of data, including text, image, and sound. Information users are surprised and their knowledge and experience are challenged as expressive methods of information visualization evolve. As a result, appropriately adding guidance or comments in the visual interface will help users understand information better. Aside from formal symbols, the design should also conform to the audience's visual experience, place the core information content in the center, and guide the reading sequence with flow symbols like arrows to improve reading efficiency.

Class perception is used to measure the perceptual strength of the color and spatial distribution of each class. For any point *p* in class *c*^*m*^, the perception degree *V*_*p*_ of this point is calculated by the following formula:

(4) $$\begin{array}{c} V_{p}=w_{p}S_{p}, \end{array}$$

where *w*_*p*_ refers to the weight of point *p* in class *c*^*m*^, and the weight is determined by the neighbor points of point *p*. *S*_*p*_ refers to the significant value of *p*. This value is obtained by formula (2). *S*_*p*_ expresses the color difference between point *p* and its surrounding neighbors.

(5) $$\begin{array}{c} S_{p}=\Delta \varepsilon \left(C_{p},\frac{1}{N_{p}}\sum_{q\in N_{p}}C_{q}\right),\\ \Delta \varepsilon \left(x,y\right)=\sqrt{\left(\Delta L^{*2}\right)+\left(\Delta a^{*2}\right)+\left(\Delta b^{*2}\right)}, \end{array}$$

where

(6) $$\begin{array}{c} \Delta L^{*}=L_{x}^{*}-L_{y}^{*},\\ \Delta a^{*}=r_{x}\cos\;\theta_{x}-r_{y}\cos\;\theta_{y},\\ \Delta b^{*}=r_{x}\sin\;\theta_{x}-r_{y}\sin\;\theta_{y}. \end{array}$$

Assuming that *X* is divided into *C* classes, and each *x*_*i*_ corresponds to a class label *I*(*x*_*i*_), then the data of class *c* are expressed as

(7) $$\begin{array}{c} \left\{X_{1}^{c},X_{2}^{c},\ldots ,X_{n}^{c}\right\}, \end{array}$$

where *n* is the number of data in the *c* class, *c* ∈ {1,2,…, *C*}. The data of different classes are divided as much as possible, and the objective function is as follows:

(8) $$\begin{array}{c} \max tr\frac{P^{T}S_{b}P}{P^{T}S_{w}P}, \end{array}$$

where *S*_*b*_ and *S*_*w*_ represent the class spacing dispersion and the intra-class distance dispersion, respectively, and the specific definitions are as follows:

(9) $$\begin{array}{c} S_{b}=\sum_{C=1}^{C}n_{c}\left(u_{c}-u\right){\left(u_{c}-u\right)}^{T},\\ S_{w}=\sum_{C=1}^{C}\sum_{i}^{n}\left(x_{i}^{c}-u_{c}\right){\left(x_{i}^{c}-u_{c}\right)}^{T}, \end{array}$$

where *u*_*c*_=∑*x*_*i*_^*c*^/*n*_*c*_ is the mean value of the *c*th data; *u* is the mean value of all data, the center point of all data.

The purpose of data analysis is to concentrate, extract, and refine a large amount of hidden information of data to find the inherent laws of the research objects, so that people can understand, judge, and make corresponding decisions and actions faster and better. On the one hand, information visualization should try to call the familiar visual features of users to construct the visual effect of information; and on the other hand, frequent visual thinking training can enrich information users' experience and knowledge stored in their brains and make visual thinking activities more efficient. In information visualization, it is not to look for symbols with specific meanings to represent, but to consider the whole information view, combine information content and context, and adopt the “proper principle” to represent with visual symbols. The modern environment provides a space for innovation and breakthrough in the design thinking and concept of visual communication design. We can make visual creation according to this selective way of reading information, so that the audience can fully participate in the whole design process, thus obtaining a more humanized visual experience.

## 4. Result Analysis and Discussion

With the progress of society, the carrier of visual information dissemination is constantly changing with the development of technology, which all affects the expression of visual information such as graphics, characters, colors, etc. in visual communication design, and also affects the change of thinking mode of design creation. In the practice of visual representation of information visualization, the construction of information model refers to the selection of appropriate organization arrangement. Visual representation design of information is a process of rational and perceptual thinking. Rational information model construction plays an important supporting role in visual representation design of information visualization. Human-computer interaction plays an important role in information visualization, and a large amount of data can only be perceived through human-computer interaction. Man-machine interaction transmits information naturally and efficiently, and allows users to get a good understanding. Good interactive mode and simple user interface can help people get relevant information quickly.  Figure 3 shows the convergence of the three algorithms as the number of iterations increases.

It can be seen that the algorithm in this article gradually converges with the increase of iteration times. This is due to the difference of objective functions of different methods. The four elements of visual design, such as text, graphics, color, and layout, are the foundation of information design, and the accurate application of them will help the accurate expression of information design. Timeliness is the main feature of dynamic visual design. From graphic design to dynamic design, the form of font design changes from a static entity to a digital virtual scene based on the concepts of time and space. Visual information from the physical world is detected visually, and then the target information is screened by visual attention mechanism, and it is decided which information needs to be processed by consciousness and which can be directly reflected. Consciousness will further process the input information, eventually forming empirical knowledge and storing it in memory for later advanced rational cognition. In order to verify the performance of this algorithm, we selected F1 value and precision as two indexes for many experiments. The experimental results of F1 value are shown in Figure 4, and the precision results are shown in Figure 5.

Systematic design method includes two processes: analysis and synthesis. Analysis precedes synthesis, and existing data information is improved after analysis to achieve new synthesis. For graphic information integration design, it is required to link the analysis and integration methods, start with the whole system, analyze and extract effective data information, and synthesize it into information visualization presentation form. In dynamic design, the development of digital technology and information technology makes it possible for the spatial attribute of characters. Time and space are two inseparable concepts in the movement. In the transformation of space, we can constantly experience the visual experience brought by movement and feel the flow of time, so as to better receive information. The interactive infographic is programmed by software such as Flash or Dreamweaver, integrates the data that have been converted into graphic language, and presents it in the form of aesthetics according to scientific data. Its presentation form is not only a moving picture, but also viewers can interact with short films on the media with their own concerns, which is more flexible than video infographics. In this chapter, several experiments are carried out to verify the feasibility and practicability of this algorithm. The experimental results of different indexes of the algorithm are shown in Table 1.

Parametric design is a term used in the design world to describe the process of establishing a specific relationship. Other elements change when one changes. Because of its various meanings and postures, each font has a unique emotional effect. Fonts are valuable due to their diverse personalities. As a result, understanding the expression of words for the transmission of information is critical in visual communication design. Consciousness will focus on dealing with new and different information, learning and adapting as a result, and the information processed by consciousness will be stored in memory as a new source of knowledge. As a result, based on visual objectives, information visualization should provide a reasonable explanation or cognitive clues to some strange and novel information, and then assist consciousness in better completing cognitive tasks.  Figure 6 depicts the effectiveness assessment of visual communication interaction design.

From the data in Figure 6, it can be seen that this design is effective and practical, which can enhance the perception of visual trajectory. Long-term memory, like a permanent box, holds a large amount of information and can extract activation information at any time. This requires a series of structures in the design process to conform to cognitive thinking and human cognitive behavior, so that the design activities can be carried out according to evidence and in the right direction. The survey results of audience demand satisfaction of visual information communication design are shown in Table 2.

The “dynamic design” in interface design has been paid more and more attention by visual design practitioners. The unique dynamic design can express the distinctive personality of the software and create fascinating effects. At the same time, it can also appease users through the use experience, so that the audience can get a relaxed and pleasant feeling when reading information, thus truly achieving humanization.  Figure 7 shows the survey results of user satisfaction with different design methods.

From the survey results of user satisfaction, it can be seen that users are more satisfied with this design method. This chapter carries out a lot of experiments and analyzes and summarizes the superiority of visual communication design in information transmission. Through research, it is found that the accuracy of this algorithm is 96.03%, and the highest evaluation of user satisfaction is 95.93%. This algorithm has faster convergence speed and greater generalization ability.

## 5. Conclusion

In the field of information visualization, visual communication design is becoming more and more involved. It is an essential component of the development of data visualization. Information visualization will develop in a more personalized and customized direction in the future, with the arrival of experience economy and the rapid development of Internet applications, and the presentation form of information visualization will not be limited to two-dimensional plane, but will pay more attention to integration with interactive experience. Through the power of images, information visualization brings dull data to life, allowing readers to grasp information quickly and leave a lasting impression. Relevant personnel should concentrate on the visualization form and mode of interaction when dealing with information visualization design. With the help of psychology and communication knowledge, this article examines the kernel of information visualization and visual representation. The audience “decodes” information through visual symbols to obtain information, according to this study. Simultaneously, it is proposed that by expounding on the concept of information visualization and analyzing the cognitive tasks and characteristics of each stage of visual communication, information users can be effectively assisted to acquire and understand information better by lowering the cost of information users in the visual thinking stage and improving their visual thinking response efficiency. Many tests show that the algorithm has a faster convergence speed and a greater ability to generalize. This algorithm has a 96.3% accuracy rating and a 95.93% user satisfaction rating. This research has certain reference value. However, due to the limitation of knowledge level and research time, there are still some problems in this article. This article is only a preliminary study of information expression, and there are still a lot of research on the details of expression and visual elements. The research of visual information interaction mode has sustainable attention and exploration significance in the future academic research and production practice and should be deeply discussed and studied.

## Figures and Tables

**Figure 1:** Information visualization process and system structure diagram.

**Figure 2:** Interactive design of visual communication based on information visualization.

**Figure 3:** Convergence of algorithm.

**Figure 4:** Experimental results of F1 value of algorithm.

**Figure 5:** Experimental results of algorithm accuracy.

**Figure 6:** Comparison of the effectiveness of visual communication interaction design.

**Figure 7:** User satisfaction results.

**Table 1:** Experimental results of each index.

Algorithm	Average absolute error	Recall rate	Accuracy rate
Grid layout algorithm	0.373	0.874	0.798
Force-guided layout algorithm	0.469	0.806	0.806
Climbing algorithm	0.327	0.769	0.884
Color optimization algorithm	0.389	0.9050.5	0.914
Feature-based tracking algorithm	0.205	0.914	0.908
Algorithm in this article	0.097	0.958	0.948

**Table 2:** Survey results of audience demand satisfaction of visual information communication design.

Index	Score (1–10)				
	1∼2(%)	3∼4(%)	5∼6 (%)	7∼8 (%)	9∼10(%)
Functionality	18.64	21.36	29.78	52.24	37.48
Cognition	17.02	20.35	49.31	46.57	42.35
Interactivity	19.93	23.64	24.57	34.32	76.61
Comprehensiveness	5.89	8.97	14.63	18.54	78.32
Accuracy	10.15	16.79	19.03	25.24	81.69
Interesting	23.69	19.63	24.35	59.37	43.57
Artistry	9.87	28.73	77.32	40.51	27.65
Novelty	17.98	37.46	20.56	18.69	19.54
Emotional expression	18.54	12.89	16.67	42.05	56.14
Color	15.57	27.99	48.51	19.79	20.06

## Data Availability

The data used to support the findings of this study are available from the author upon request.
